# Cellular and Synaptic Mechanisms That Differentiate Mitral Cells and Superficial Tufted Cells Into Parallel Output Channels in the Olfactory Bulb

**DOI:** 10.3389/fncel.2020.614377

**Published:** 2020-12-22

**Authors:** Shelly Jones, Joel Zylberberg, Nathan Schoppa

**Affiliations:** ^1^Department of Physiology and Biophysics, University of Colorado Anschutz Medical Campus, Aurora, CO, United States; ^2^Department of Physics and Center for Vision Research, York University, Toronto, ON, Canada

**Keywords:** olfaction, olfactory bulb, mitral cell, tufted cell, parallel pathways

## Abstract

A common feature of the primary processing structures of sensory systems is the presence of parallel output “channels” that convey different information about a stimulus. In the mammalian olfactory bulb, this is reflected in the mitral cells (MCs) and tufted cells (TCs) that have differing sensitivities to odors, with TCs being more sensitive than MCs. In this study, we examined potential mechanisms underlying the different responses of MCs vs. TCs. For TCs, we focused on superficial TCs (sTCs), which are a population of output TCs that reside in the superficial-most portion of the external plexiform layer, along with external tufted cells (eTCs), which are glutamatergic interneurons in the glomerular layer. Using whole-cell patch-clamp recordings in mouse bulb slices, we first measured excitatory currents in MCs, sTCs, and eTCs following olfactory sensory neuron (OSN) stimulation, separating the responses into a fast, monosynaptic component reflecting direct inputs from OSNs and a prolonged component partially reflecting eTC-mediated feedforward excitation. Responses were measured to a wide range of OSN stimulation intensities, simulating the different levels of OSN activity that would be expected to be produced by varying odor concentrations *in vivo*. Over a range of stimulation intensities, we found that the monosynaptic current varied significantly between the cell types, in the order of eTC > sTC > MC. The prolonged component was smaller in sTCs vs. both MCs and eTCs. sTCs also had much higher whole-cell input resistances than MCs, reflecting their smaller size and greater membrane resistivity. To evaluate how these different electrophysiological aspects contributed to spiking of the output MCs and sTCs, we used computational modeling. By exchanging the different cell properties in our modeled MCs and sTCs, we could evaluate each property's contribution to spiking differences between these cell types. This analysis suggested that the higher sensitivity of spiking in sTCs vs. MCs reflected both their larger monosynaptic OSN signal as well as their higher input resistance, while their smaller prolonged currents had a modest opposing effect. Taken together, our results indicate that both synaptic and intrinsic cellular features contribute to the production of parallel output channels in the olfactory bulb.

## Introduction

In many sensory systems, the brain structure that is involved in the initial processing of information is endowed with multiple types of output cells that carry different types of information about the stimulus. One example is in vision, where the many types of retinal ganglion cells (RGCs) create parallel pathways from the retina to the Lateral Geniculate Nucleus (LGN). The diversity of RGCs is theorized to increase the sensitivity of the retina to a wider range of inputs (Baden et al., 2016). The primary processing structure for olfaction, the olfactory bulb, also appears to have multiple output neurons, in the form of mitral cells (MCs) and different subpopulations of tufted cells (TCs). Recent physiological studies indicate that MCs and TCs have markedly different responses to odors. MCs require greater concentrations of odorant to be activated, displaying rightward-shifted odor-concentration vs. response “activation” curves, and have a much narrower odor tuning profile (Nagayama et al., 2004; Griff et al., 2008; Fukunaga et al., 2012; Igarashi et al., 2012; Kikuta et al., 2013). MCs and TCs also differ in their anatomical projections. TCs display selective projections to the anterior olfactory nucleus and the olfactory tubercle, while MCs project to the piriform cortex in addition to these regions (Nagayama et al., 2010; Igarashi et al., 2012). Thus, MCs and TCs appear to convey distinct information about an odorant stimulus and send it to overlapping but not identical, cortical areas.

Despite evidence for different sensitivities to odorants for MCs and TCs, the mechanisms underlying these differences are unresolved. In one study comparing the responses of MCs and TCs to afferent stimulation conducted in brain slices, Burton and Urban (2014) suggested that the greater sensitivity of TCs might be explained by both stronger direct monosynaptic signals from olfactory sensory neurons (OSNs) as well as greater intrinsic excitability of TCs vs. MCs. The greater intrinsic excitability may reflect the smaller size of TCs (Macrides and Schneider, 1982; Orona et al., 1984) and the associated greater whole cell input resistance (Hamilton et al., 2005; Antal et al., 2006; Burton and Urban, 2014). These mechanistic studies however had a number of limitations, including the fact that the analysis was confined mainly to a subclass of TCs, the middle tufted cells (mTCs), with cell bodies located in relatively deep portions of the external plexiform layer (EPL). Output TCs also include superficial TCs (sTCs), which have different cell sizes and apical dendrite lengths vs. mTCs (Macrides and Schneider, 1982; Mori et al., 1983; Orona et al., 1984; Mori, 1987) and also appear to have very different sensitivities to odor (Griff et al., 2008). In addition, the responses of each MC/TC in prior mechanistic studies were generally analyzed at only a single OSN stimulation intensity. This makes it more difficult to draw definitive conclusions about the mechanisms that underlie *in vivo* properties such as MCs' rightward-shifted activation curves measured in response to a range of odor concentrations (Igarashi et al., 2012; Kikuta et al., 2013).

A last point of uncertainty reflects the contribution toward spiking of excitatory current components that are distinct from monosynaptic OSN inputs. Within MCs, OSN stimulation elicits prolonged currents that include both feedforward excitation derived from a class of excitatory interneurons known as external tufted cells (eTCs, distinct from output sTCs and mTCs; De Saint Jan et al., 2009; Najac et al., 2011; Gire et al., 2012) along with an additional sustained current mediated by Group I metabotropic glutamate receptors (mGluRs; Schoppa and Westbrook, 2001; Heinbockel et al., 2004; Ennis et al., 2006; Yuan and Knöpfel, 2006; De Saint Jan and Westbrook, 2007). These prolonged current components account for a large majority of the excitatory charge in MCs (Gire et al., 2012; Vaaga and Westbrook, 2016) but remain largely uncharacterized in TCs.

Here, we used whole-cell patch-clamp recordings in mouse olfactory bulb slices and computational modeling to examine the mechanisms that contribute to differences in responsiveness of MCs and output TCs to afferent stimulation. For the sake of consistency, our analysis of output TCs was focused on one subclass, the sTCs with cell bodies located in the most superficial region of the EPL. sTCs are the most morphologically distinct from MCs of all output TCs, with the shortest apical dendrites and limited lateral dendrites, and also appear to be the most physiological distinct from MCs (Griff et al., 2008). Our broad strategy was first to characterize the different excitatory current components and intrinsic properties of MCs and sTCs experimentally across widely varying OSN stimulation intensities and then use computational models to test the respective contribution of the different properties to potential differences in the cells' spiking. In the experimental section of the study, we also compared MC and sTC responses to those of eTCs. eTCs have been better characterized than sTCs (Hayar et al., 2004a,b; Antal et al., 2006; De Saint Jan et al., 2009; Najac et al., 2011; Gire et al., 2012; Vaaga and Westbrook, 2016), but not using widely varying OSN stimuli nor with respect to their prolonged current components.

## Methods

### Experimental Animals

All experiments were approved by the Institutional Animal Care and Use Committee at the University of Colorado Anschutz Medical Campus. Data are from C57BL/6 mice (Charles River, Wilmington, MA, USA) at postnatal age 13–26 days, of both sexes. While housed in the UCAMC facility, mice had full, and continuous access to food and water.

### Electrophysiological Recordings in Mouse OB Slices

Horizontal slices (300–400 μm) were prepared from OBs of mice following general isoflurane anesthesia and decapitation, as described previously (Pouille et al., 2017). Bulb slices were visualized using an upright Axioskop 2FS microscope (Carl Zeiss) with differential interference contrast optics video microscopy and a CCD camera. Cells were visualized with a 40X water-immersion objective. All experiments were performed at 29–34°C.

The base extracellular recording solution contained the following (in mM): 125 NaCl, 25 NaHCO_3_, 1.25 NaH_2_PO_4_, 25 glucose, 3 KCl, 2 CaCl_2_, 1 MgCl_2_, pH 7.3, and was oxygenated (95% O2, 5% CO_2_). Patch pipettes for whole-cell recordings (4–8 MΩ) contained 125 K-gluconate, 2MgCl_2_, 0.025 CaCl_2_, 1 EGTA, 2 NaATP, 0.5 NaGTP, 10 HEPES, pH 7.3 with KOH. The sodium channel blocker QX-314 (10 mM) was included to block action potential firing. Current and voltage signals were recorded with a Multiclamp 700A amplifier (Molecular Devices), low-pass filtered at 1–2 kHz, and digitized at 10 kHz. The reported value for the holding potential for our excitatory current measurements (−77 mV) has been corrected for a liquid junction potential. OSN stimulation was performed by placing a broken-tip patch pipette (10 μm diameter) in the ON layer, ~50 μm superficial to the target glomerulus of the test cell. Brief pulses (100 μs) triggered by a stimulus isolation unit were applied, with an interstimulus interval of 20 s. Data were acquired using AxographX. Morphological analysis of the cells, including determination of target glomeruli, was done for whole-cell recordings by including Alexa 488 (100 μM) in the patch pipette. Selected cells had apical dendrites targeted to glomeruli at the slice surface, which facilitated stimulation of OSNs at target glomeruli.

Cell types were defined based on several criteria, as described previously (Pinching and Powell, 1971; Hayar et al., 2004a; Gire and Schoppa, 2009; Gire et al., 2012). Mitral cells (MCs) had somas located in the mitral cell layer. External tufted cells (eTCs) had an ellipsoid-shaped cell body (diameter, 10 μm) in the glomerular layer, no lateral dendrites, and apical dendrites that filled target glomeruli. Superficial tufted cells (sTCs) had cell bodies that were located in the outer third of the external plexiform layer, had at least one lateral dendrite, and a single apical dendrite that filled target glomeruli. Nomenclature around tufted cell subtypes has been somewhat confusing in the field. Our sTCs likely correspond to the class of “eTCs” described by Antal et al. (2006) that had lateral dendrites; the sTCs are also the “superficial middle tufted” cells of Gire et al. (2012).

In our measurements of excitatory currents, care was taken to perform voltage-clamp recordings using a holding potential (−77 mV) that was near the reversal potential for chloride for our experiments (−89 mV). This should have minimized the contribution of potentially contaminating GABA_A_ receptor-mediated currents. In principle, another strategy to eliminate such currents woul have been to use a GABA_A_ receptor blocker. However, prior studies have shown that such blockers cause large increases in prolonged excitatory currents in MCs that are evoked by OSN stimulation (Carlson et al., 2000; Schoppa and Westbrook, 2001). This is because at least part of the slow current reflects feedforward excitation from eTCs whose activity can be impacted by inhibition. Thus, while blockade of GABA_A_ receptors may have added greater certainty that the recorded currents did not include a small contaminating GABAergic current, it would have introduced what we believe is a significantly worse problem in interpreting the slow currents.

### Analysis of Electrophysiological Recordings

In the analysis of EPSCs evoked by OSN stimulation, the peak of the OSN-EPSC was defined as the maximum current response within 6 ms of stimulus onset. Peak OSN values that were plotted as a function of OSN stimulation intensity were fitted to a sigmoidal function:

(1) $$\begin{array}{r} y=\frac{\left(a1-a2\right)}{1+e^{\frac{x-x_{0}}{dx}}}+a2 \end{array}$$

with *a2* was defined as the maximum response, *x* was the OSN stimulation intensity, *x*_0_ was the *stimulus*_50*%max*_ or the stimulus necessary to elicit half of the maximum response, *dx* was the steepness of the sigmoidal curve, and *a1* was the minimum response.

In the estimates of unitary EPSCs (uEPSCs), a minimum stimulus intensity was found that produced a response in <50% of trials, for at least 10 trials. We then measured the amplitude of the unitary EPSC by taking the average amplitude over 1.5 ms of each uEPSC event, centered on the time frame with the largest current response. Spontaneous EPSCs (sEPSCs) were found using an event detection search in AxographX. The amplitudes were measured with the same methodology as the uEPSC amplitudes.

In the analysis of the prolonged current components, estimates of its magnitude were obtained by integrating the current measured 6–300 ms after stimulation. In most cells, the decay of the OSN-EPSC appeared to be complete by 6 ms after the stimulus. We also measured the amplitude of the current at 300 ms after stimulus by taking the average current over 1 ms.

### Neuron Modeling

Simulations of excitatory currents and spiking behavior in MCs and sTCs were performed using NEURON (Hines and Carnevale, 1997). The morphology of the MC model was based on the morphology of MCs from Migliore et al. (2005). For the sTC, we used a soma 25% of the area of the MC soma, an apical dendrite 30% of the length of the MC apical dendrite, and lateral dendrites with 50% of the total lateral dendrite length as compared to MCs. The apical dendrite length for sTCs was based on our own morphological measurements of sTCs and MCs, wherein we found that the length of sTC apical dendrites (mean ± SE of trunk length = 58 ± 6 μm, *n* = 11) was ~29% that of MCs (mean ± SE of trunk length = 206 ± 16 μm, *n* = 6). The values for the relative size of the sTC soma and lateral dendrites were based on values reported for sTC reconstructions (Tavakoli et al., 2018) vs. those reported for MCs (Burton and Urban, 2014), with some modest deviations (see below). For modeling the passive membrane properties and active conductances of each cell, we used membrane parameters that were similar to Bhalla and Bower's MC (Bhalla and Bower, 1993). The only difference between the cells' ion channel parameters was the density of the leak channels. For each cell, the density was chosen to correspond to the resistance per unit area value that we estimated based on the cell's measured whole-cell input resistance (see Table 1). In the calculations of resistance per unit area, we assumed that each MC or each sTC had the same membrane surface area; this value was calculated based on the morphology of the model MC or sTC. We used the published resting potentials for MCs and TCs from Burton and Urban (2014).

**Table 1:** Intrinsic properties of MCs and sTCs that were used in the simulations.

**Cell Type**	**R_**input**_ (MΩ)**	**Surface area (μm^**2**^)**	**Resistance per unit area (Ωcm^**2**^)**	**V_**rest**_ (mV)**
MC	87.4 ± 4.3 (*n* = 8)	4,010	3500 ± 200 (*n* = 8)	−54
sTC	447.3 ± 28.6 (*n* = 7)	1,860	8300 ± 500 (*n* = 7)	−56

*Parameters included the whole-cell input resistance (R_input_) experimentally measured across our test cells, the surface area of the model cell (see Methods), membrane resistivity (resistance per unit area) derived from R_input_ and morphological parameters, and cell resting potential (V_rest_). Resting potential values were taken from the analysis of MCs and TCs in Burton and Urban (2014)*.

In terms of inputs into the model cells, three types of excitatory conductances were applied to the distal end of the dendritic tuft branches to match the recorded excitatory currents. These included a rapid OSN-EPSC, a slower transient current with decay kinetics of ~50–100 ms, and a step current. The latter two may have, respectively, reflected the feed-forward excitation mediated by eTCs (De Saint Jan et al., 2009; Najac et al., 2011; Gire et al., 2012) and a more sustained current mediated by activation of Group I mGluRs (Schoppa and Westbrook, 2001; Heinbockel et al., 2004; Ennis et al., 2006; Yuan and Knöpfel, 2006; De Saint Jan and Westbrook, 2007). For the OSN-EPSC and transient prolonged current, we used the kinetics from our recorded excitatory current for each synapse. Appropriate peak amplitudes for the input conductances were found using the voltage-clamp feature of NEURON. Using a binary search method, conductance amplitudes were varied until the amplitude of the simulated current response was within 10% of the experimentally observed current response. This approach enabled us to estimate the synaptic input at the distal dendrites that would give rise to the observed excitatory current recorded at the cell soma.

The MC and sTC models were first used to estimate the spiking properties of MC/sTCs at different OSN stimulation intensities. The spiking properties (number of spikes and spike probability) were determined for each cell and at each OSN stimulation intensity based on three trials of experimentally recorded current at each stimulation intensity that were input into the model cell. This procedure applied over our population of test MCs and sTCs enabled us to accumulate statistics about the spike responses of each cell type. An estimate of the stimulus-response relationship for each MC and sTC was obtained by fitting a sigmoidal function (see Eqtn 1 above) to the relationship between stimulation intensity and the number of spikes for each cell (see **Figure 4F**).

An exchange procedure in NEURON was used to estimate the contribution of each of three cellular properties to the sTC/MC spike response. The properties exchanged included the OSN-EPSC, the prolonged current, and the intrinsic cell properties. When the prolonged current was exchanged, we grouped the slow transient and step current together as one component. For the intrinsic property substitution, we grouped cell morphology, cell resting potential, and resistance per unit area to be a single component to be exchanged at once. Whether the exchange of a particular cellular property induced a statistically significant change in spike number at a given OSN stimulation intensity was determined through the following procedure, as described here for substituting the OSN-EPSC of the sTC into the MCs. We first determined a Mann-Whitney U statistic for each MC by comparing the number of spikes across three experimental trials in the intact version of that MC (with its “native” OSN-EPSC) with the number of spikes in that MC with an OSN-EPSC substituted in that reflected the corresponding trials in all sTCs. Because there were seven test sTCs and three trials were recorded per sTC, this per-MC statistical analysis involved comparing 21 spike number values representing substituted OSN-EPSCs from the sTCs to three spike number values in the native MC (representing its three experimental trials). We then combined the Mann-Whitney U results for each MC (*n*_*MC*_ = 8) with a Fisher Combined Test to determine the statistical significance of the difference in MC responses caused by substituting the OSN-EPSC.

Some of the morphological parameters that were used for sTCs in the simulations (see above) differed modestly from the mean values reported for sTCs by Tavakoli et al. (2018). For example, the 25% cell soma area was slightly smaller than the reported soma areas for sTCs in that study, which, depending in the subtype of sTCs, were 28 or 31% of the value for MCs (Burton and Urban, 2014). To confirm that the slightly smaller cell soma did not impact our results, we repeated the simulations of spiking in one sTC (control, unswapped condition) using a soma area that was 31% (rather than 25%) that of MCs, finding that, across all trials and all stimulation intensities, the number of simulated spikes did not change (mean = 8.3 spikes with soma 25 and 31% that of MCs). A value for the lateral dendritic length for sTCs that is 50% that of MCs was likely on the high end of a range of possible lengths. Tavakoli and co-workers reported values for the lateral dendritic volume for sTCs (mean ± SD = 1062 ± 941 μm) that are about one-third of those reported for MCs (mean ± SD = 3434 ± 2221; Burton and Urban, 2014); differences between lateral dendritic volume also appear to scale linearly with differences in length (Burton and Urban, 2014). When we simulated sTCs with a lateral dendritic length that was 33% (rather than 50%) of that of MCs, we found that the mean value of simulated spikes increased modestly (from 8.3 to 10.5; in the same sTC as above). The greater number of spikes was expected since reducing the lateral dendrite size decreased the total size of the model sTC. The fact that most of our simulations used a longer lateral dendrite for sTCs suggested that our analysis, if anything, was conservative, underestimating spike sensitivity differences between sTCs and MCs.

### Sensitivity Measurements

This analysis compared the sensitivity of a population of bulbar output cells under two conditions, Condition A, when the population included MCs and sTCs with distinct relationships between OSN stimulation intensity and spike number (the actual situation), and Condition B in which the cells had properties that were the average (“hybrid”) between that of MCs and sTCs. The stimulus-response behavior of any one cell was defined by the sigmoidal curve fitted to the simulated OSN stimulation vs. spike number data for that cell (**Figure 4F**). The sensitivity of spiking to changes in OSN stimulation intensity for each cell was then defined by the squared derivative of the fitted sigmoidal function at every stimulus intensity.

For Condition A, we wished to remove the contribution to the sensitivity measurement of the variability of spiking behavior amongst the cells within a subgroup (MCs or sTCs). Hence, the stimulus response curve for each cell within a subgroup was the average of the fitted sigmoidal curves for that group (the red and blue curves shown in **Figure 6A**). The overall sensitivity measure for the cell population in Condition A (purple curve in **Figure 6B**) was the average of the squared derivatives for MCs and sTCs, weighted by the number of cells in each subgroup (*n*_*MC*_ = 8; *n*_*sTC*_ = 7). For Condition B, the overall sensitivity measure (black curve in **Figure 6B**) was the squared derivative of the stimulus response relationship of the average hybrid MC/sTC (black curve in **Figure 6A**).

This type of analysis would often use Fisher Information as a measure of neuronal sensitivity. Fisher Information is the signal to noise ratio obtained by dividing a sensitivity measure by the trial-to-trial variance in neuronal activities (Paradiso, 1988; Brunel and Nadal, 1998). However, due to our low number of trials per cell per stimulus intensity (three) and the nature of our stimulus (short, relatively high intensity electrical pulses), any measure of variance in our analysis was strongly underpowered. We thus could not reliably determine the Fisher Information, and instead used the squared derivative of the stimulus-response curves as a neuronal sensitivity measure.

### Statistical Analyses

Statistical significance was determined via Mann-Whitney *U* tests, except where specified otherwise. For some analyses, such as when cell properties were exchanged in NEURON, a Fisher Combined Test was used to combine the Mann-Whitney U *p*-values from all MCs.

Data values are reported as means ± SE. The asterisks in the figures generally indicate statistical significance at *p* < 0.05, except when a Bonferroni correction for multiple comparisons was applied.

### Access to Data

Our modeling results will be made available at the time of publication in ModelDB (https://senselab.med.yale.edu/modeldb/). Files to be included in ModelDB will be the hoc files with the morphologies of the model MC and sTCs, mod files that specify the intrinsic properties and excitatory conductances (OSN and prolonged), example current recordings, and binary search python files that can reproduce the example traces in **Figures 4Aii,v,B,C**. These files can also be used to fit other current recordings with excitatory conductances and convert simulated conductances into voltage traces and spiking activity. We will also include hoc and mod files with pre-fitted conductances to reproduce the traces in **Figures 5C,D**. All other raw experimental data supporting the conclusions of this article will be made available upon request by the authors, without undue reservation.

## Results

### sTCs Have Monosynaptic EPSCs That Are Smaller Than eTCs but Larger Than MCs

To compare the level of direct OSN signaling onto MCs, sTCs, and eTCs, we recorded excitatory currents in voltage-clamped cells (*V*_*hold*_ = −77 mV) in response to electrical stimulation of OSN fibers in mouse OB slices. Cell types were determined based on their location in the bulb (Figure 1Ai) as well as their morphology (Figure 1Aii; see Methods). To find the originating glomerulus of the test cells, we filled the patched cell with fluorescent dye (Alexa 488, 100 μM) and traced the cell back to the glomerulus. We then selectively recorded from cells with apical dendritic tufts located at the surface of the OB slice. This made our OSN fiber stimulation more consistent between recordings from different glomeruli and slices. The recorded current in every example of each cell type (*n*_*MC*_ = 10, *n*_*eTC*_ = 11, *n*_*sTC*_= 13) included a component that occurred with a short onset delay (≤ 2 ms) and fast rise time, consistent with it being the monosynaptic EPSC reflecting direct transmission from OSNs (the “OSN-EPSC”; see MC example in Figure 1B). In addition, all cells also displayed a distinct prolonged excitatory current component. Studies in MCs have suggested that much of this slower current reflects feedforward excitation mediated by eTCs (De Saint Jan et al., 2009; Najac et al., 2011; Gire et al., 2012).

**Figure 1:** Olfactory bulb anatomy and analysis of monosynaptic OSN-EPSCs in MCs, sTCs, and eTCs. **(Ai)** Illustration of morphology and anatomy of external tufted cells (eTCs), superficial tufted cells (sTCs), middle tufted cells (mTCs), and mitral cells (MCs) in the olfactory bulb (OB). Cells are organized within the glomerular layer (GL), external plexiform layer (EPL), and mitral cell layer (MCL). Input to the GL is from the olfactory nerve layer (ONL). **(Aii)** Images of Alexa-488-filled eTC, sTC and MC, highlighting their different morphologies. Note the different length apical dendrite in each cell-type and the presence (sTC and MC) or absence (eTC) of lateral dendrites. **(B)** Example of MC excitatory current trace in response to OSN stimulation (100 μA), recorded at a holding potential of −77 mV. The monosynaptic OSN-EPSC and prolonged current components are indicated. **(C)** Examples of excitatory currents measured in response to different stimuli (30, 50, 100, and 200 μA) from MC **(i)**, sTC **(ii)**, and eTC **(iii)**. Traces are averages of 3 trials at each stimulation level. **(D)** Peak OSN-EPSC as a function of stimulus intensity for the experiment in **(C)** with fits of a sigmoidal curve (see Equation 1 in Methods) overlaid for MC **(i)**, sTC **(ii)**, and eTC **(iii)**. Each data point reflects the current recorded in a single trial. **(E)** Peak OSN-EPSC as a function of stimulus intensity for MCs (**i**; *n* = 10), sTCs (**ii**; *n* = 13), and eTCs (**iii**; *n* = 11). Each data point is the average of three trials for each cell at each stimulation intensity. Lines connect values for the same cell. **(F)** The maximal OSN-EPSC, *OSN-EPSC*_*max*_, for each cell, grouped by cell type. Horizontal lines show the mean over cells of a given type.

To evaluate the properties of direct OSN signaling in the different cell types, we recorded the currents in each cell in response to a wide range of stimulus intensities applied to OSNs (Figure 1C) and plotted the peak amplitude of the OSN-EPSC amplitude as a function of stimulation intensity (Figures 1D,E). We then fitted the stimulus-response data for each cell with a sigmoidal function (see Methods, Equation 1) and extracted two parameters: the maximal OSN-EPSC amplitude (*OSN-EPSC*_*max*_) and the stimulus intensity needed to reach 50% of this maximum (*stimulus*_50*%max*_). In terms of *OSN-EPSC*_*max*_, eTCs had much larger values (1,283 ± 51 pA, *n* = 11) than sTCs (542 ± 16 pA, *n* = 13; *p* = 0.0002, Mann-Whitney U test) or MCs (270 ± 12 pA, *n* = 10; *p* = 0.0001, Mann-Whitney *U* test; Figure 1F). Moreover, *OSN-EPSC*_*max*_ in sTCs was a factor of two larger than *OSN-EPSC*_*max*_ in MCs (*p* = 0.0100, Mann-Whitney *U* test). *OSN-EPSC*_*max*_ at high intensities should reflect the current arising from the activation of all OSN axons that targeted the test cell. Hence, differences in *OSN-EPSC*_*max*_ between cell types should reflect differences in the current produced when all such OSN axons were activated. Importantly, the amplitudes of each cell's OSN-EPSC appeared to saturate or nearly saturate at high stimulation intensities (Figure 1E), suggesting that we were successful in our experiments at activating nearly all OSN axons that terminated on the test cells.

In the analysis of *stimulus*_50*%max*_, we found that MCs (80 ± 5 μA) and sTCs (84 ± 4 μA) had similar values (*p* = 0.93, Mann-Whitney *U* test, data not shown), consistent with the cells receiving input from populations of OSN axons with similar spatial distributions and levels of excitability. We found somewhat smaller values for *stimulus*_50*%max*_ for eTCs (42 ± 2 μA; *p* = 0.037, *p* = 0.062, in comparison with sTCs and MCs, respectively, Mann-Whitney *U* tests). We were careful not to over-interpret this difference however since the leftward shift in the stimulus-response relationship for eTCs could have reflected series resistance errors generated by the very large OSN-EPSCs in eTCs (since the errors would have most impacted the largest currents).

### Unitary EPSCs in eTCs Are Much Larger Than in MCs or sTCs

Our analysis thus far has shown that MCs, sTCs, and eTCs display substantial differences in *OSN-EPSC*_*max*_produced by stimulation of all (or nearly all) OSN axons at a given glomerulus. The different values for *OSN-EPSC*_*max*_ in MCs, sTCs, and eTCs could be explained by differences in the number of OSN axons that target the cells or differences in the current produced by each single OSN axon. To disambiguate between these possibilities, we used two approaches, the first of which was to record currents at “minimal” stimulus intensities, when current responses were produced in <50% of the trials (Figures 2A,B). The “unitary” EPSCs (uEPSCs) recorded under this condition should reflect the current arising from a single OSN axon. We found that eTCs had much larger uEPSCs (115 ± 9 pA, *n* = 6) than either MCs (25 ± 1 pA, *n* = 6; *p* = 0.0022, Mann-Whitney U test) or sTCs (32 ± 4 pA, *n* = 6; *p* = 0.0043, Mann-Whitney *U* test; Figure 2D). Interestingly, the difference in the size of the uEPSCs between eTCs and MCs/sTCs, ~4-fold, was roughly similar to the differences in *OSN-EPSC*_*max*_ in MCs, sTCs, and eTCs (see above), suggesting that larger currents generated by single OSN axons are a major factor underlying the larger *OSN-EPSC*_*max*_ in eTCs vs. MCs/sTCs. That the single OSN axon current is much larger in eTCs than MCs/sTCs was also supported by recordings of spontaneous EPSCs (sEPSCs) that were conducted in parallel (Figure 2C). sEPSCs arise in part from action potential firing in single OSN axons, and hence provide an independent estimate of the single OSN axon current (sEPSCs also reflect spontaneous release events at single synapses). eTCs had larger sEPSCs (36 ± 1 pA, *n* = 11) than sTCs (24 ± 1 pA, *n* = 13; *p* = 0.0005, Mann-Whitney U test) or MCs (19 ± 1 pA, *n* = 10, *p* = 0.0004, Mann-Whitney *U* test; Figure 2Ei). sEPSCs were also much more frequently detected in eTCs vs. MCs or sTCs (Figure 2Eii).

**Figure 2:** eTCs have larger OSN-EPSCs produced by single OSN axons than MCs or sTCs. **(A)** Example current recordings in a MC **(i)**, sTC **(ii)**, or eTC **(iii)** made in response to OSN stimulation under minimal stimulus conditions, when the response failure rate was ≥50%. Stimulation intensities were 10.8 μA (MC), 20 μA (sTC), or 18 μA (eTC). Multiple trials are overlaid for each cell: 27 (MC), 23 (sTC), 21 (eTC). **(Bi,ii,iii)** Peak current amplitudes for the experiments in **(A)**. Each data point reflects a single trial. **(C)** Current recordings in a MC **(i)**, sTC **(ii)**, or eTC **(iii)** made in the absence of stimulation (*V*_*hold*_ = −77 mV). Inward current deflections reflect spontaneous EPSCs (sEPSCs). **(D)** Average unitary EPSC amplitudes for each cell, grouped by cell type. **(E)** Average sEPSC amplitude **(i)** and frequency **(ii)** for each cell, grouped by cell type.

Comparing sTCs and MCs, we did not observe a significant difference in the size of either the uEPSCs nor the sEPSCs (*p*_*uEPSC*_ = 1.0, *p*_*sEPSC*_ = 0.270, Mann-Whitney *U* tests). This was distinct from the *OSN-EPSC*_*max*_values, which were ~2-fold larger in sTCs than in MCs (see above). One interpretation of these data is that sTCs and MCs have similar sized currents arising from stimulation of single OSN axons but sTCs have more convergent axons than MCs. However, we caution against such an interpretation because the small size of the uEPSCs/sEPSCs in MCs/sTCs meant that we were generally operating at the limits of our experimental detection capabilities. That the average sEPSC in MCs was likely to be much smaller than our reported values was also supported by the extremely low frequency of sEPSCs in MCs (0.09 ± 0.01 Hz, *n* = 10; Figure 2Eii). This suggested that we likely were missing a large fraction of small sEPSCs in MCs in our spontaneous event detection.

### Characteristics of the Prolonged Current Components in MCs, sTCs, and eTCs

Prior studies have provided evidence that most of the excitatory current in MCs that is evoked by OSN stimulation (in terms of charge contribution) is not the rapid monosynaptic EPSC but rather a prolonged current that in part reflects feedforward excitation mediated by eTCs (De Saint Jan et al., 2009; Najac et al., 2011; Gire et al., 2012; Vaaga and Westbrook, 2016). Activation of Group I mGluRs also contributes to a more prolonged depolarizing current in MCs (Schoppa and Westbrook, 2001; Heinbockel et al., 2004; Ennis et al., 2006; Yuan and Knöpfel, 2006; De Saint Jan and Westbrook, 2007) that could be due to glutamate release from OSNs or eTCs. We thus wondered whether the properties of the prolonged currents also differed between the different cell types. In our analysis, we found that OSN stimulation evoked prolonged currents (longer-lasting than the monosynaptic EPSC) in all cell types (Figure 3A). In some cells and at some stimulation intensities, the prolonged currents had two distinct components, one with a duration of ~50 ms and a second that was sustained for hundreds of milliseconds. However, not all cells displayed these distinct components, and, for ease of analysis, we did not separate the prolonged current into different components.

**Figure 3:** sTCs have smaller prolonged currents than MCs or eTCs. **(A)** Example traces of MC, sTC, and eTC current responses to OSN stimulation (100 μA), expanded and overlaid to highlight differences in the prolonged currents. Note the significant current that persists out to 300 ms after stimulation in the MC and eTC but not the sTC. **(B)** Integrated prolonged current response (6–300 ms after stimulus) for MCs, sTCs, and eTCs. Each data point reflects the average of three stimulus trials in a single cell. **(C)** Amplitude of current response of MCs, sTCs, and eTCs measured 300 ms after OSN stimulation. Each data point reflects the average of three stimulus trials in a single cell. Note the larger sustained current in MCs and eTCs than in sTCs at the higher stimulation intensities.

We first compared the size of the prolonged currents by integrating the charge in a window (6–300 ms) after OSN stimulation that should have mainly excluded the OSN-EPSC. Across cell-types and stimulation intensities, the most consistent observation was that the prolonged current was smaller in sTCs than in MCs or eTCs (Figure 3B). The current in sTCs was significantly smaller than that of eTCs at all stimulation intensities (e.g., at 100 μA, sTCs: 11.6 ± 3.2 pC, *n*_*sTC*_ = 13; eTCs: 29.1 ± 4.6, *n*_*eTC*_ = 11; *p* = 0.0016, Mann-Whitney *U* test) and smaller than that of MCs at 100 μA (MCs: 18.9 ± 4.3 pC, *n*_*MC*_ = 10; *p* = 0.0498, Mann-Whitney *U* test). The prolonged currents were also somewhat larger in eTCs vs. MCs at 100 μA stimulation (*p* = 0.0378).

Direct visualization of the data traces in Figure 3A suggested that the larger integrated charge values for MCs and eTCs vs. sTCs in the prolonged current analysis could have reflected at least in part a difference in the sustained current. We quantified this difference by measuring the current amplitudes at 300 ms post-stimulus, finding that the current in MCs was indeed much larger than that of sTCs at both 100 μA (MCs: 52 ± 15 pA, *n*_*MC*_= 10; sTCs: 27 ± 10 pA, *n*_*sTC*_ = 13; *p* = 0.028, Mann-Whitney *U* test) and 200 μA (MCs: 77 ± 19 pA; sTCs: 2 ± 2 pA; *p* < 0.0001, Mann-Whitney *U* test). eTCs also had much a larger sustained current than sTCs at 200 μA (eTCs: 81 ± 19 pA; *p* < 0.0001 in comparisons with sTCs, Mann-Whitney *U* test). These results indicate that sTCs are unique in not having a large sustained current at high OSN stimulation intensities.

### sTCs Display Higher Spike Probability and Spike Number Than MCs in Simulated Spike Responses

We next set out to understand how the *in vitro* current response to OSN stimulation relates to the spike responses of the output neurons of the bulb. For this comparison, we focused our analysis on MCs and sTCs, since eTCs are not output neurons, and there have been no *in vivo* characterizations of eTCs (as we have defined them; see Methods). Our strategy, as outlined in Figure 4A, was to use a modeling approach in NEURON software (Bhalla and Bower, 1993; Hines and Carnevale, 1997; Migliore et al., 2005), where we simulated spike responses in a modeled cell that received the experimentally observed excitatory currents. For each individual cell and for each of four OSN stimulation intensities, this procedure was repeated for three experimental trials (Figures 4B,C) so that statistics about the responses of MCs and sTCs could be accumulated. This approach was preferred vs. direct recordings of spiking in MCs and sTCs, since, in our subsequent analysis (see below), we exploited the modeling to exchange the different excitatory current components in the two cell types. This enabled us to determine their respective contributions to spike differences between MCs and sTCs. In each simulation, we took care to match the MC and sTC models to the known cellular morphology, resting membrane potential, and ion channel types and densities (see Methods and Table 1). Our simulations also took into account the input resistances of each individual cell determined experimentally by adjusting the values for the membrane resistance per unit areas in the model cells. Values for the whole-cell input resistance were on average ~5-fold larger in sTCs than in MCs (MCs: 87 ± 4 MΩ, *n* = 8; sTC: 447 ± 29 MΩ, *n* = 7; *p* = 0.0001, Mann-Whitney *U* test).

**Figure 4:** Simulated spiking behavior in MCs and sTCs. **(A)** Method of simulating voltage responses based on experimental recordings of excitatory currents. **(i)** Example recording of excitatory current in a MC in response to OSN stimulation (50 μA). **(ii)** An excitatory current produced by NEURON simulated to match the experimental recording in part **(i)**. The trace was generated by inputting synapses onto the distal dendrite of the model MC and varying the amplitude of the synaptic conductances until the simulated current matched the experimental trace. **(iii,iv)** Deconstruction of the simulated excitatory current in part **(ii)** into a monosynaptic OSN-EPSC and a prolonged current. The prolonged current itself reflected the sum of two components, a transient “feedforward” excitatory component and a step current. **(v)** One trial of simulated voltage in the model MC receiving the current in part **(ii)**. **(B)** Examples of simulated MC voltage traces in response to 30 **(i)** and 100 μA **(ii)** OSN stimulation. Three trials are shown at each stimulation intensity, corresponding to three trials of experimentally recorded currents. **(C)** Examples of simulated sTC voltage traces in response to 30 **(i)** and 100 μA **(ii)** OSN stimulation. **(D)** Summary of the number of simulated spikes at different stimulus intensities in modeled MCs and sTCs. Each data point reflects the average of three experimental trials in a single cell. **(E)** Summary of the probability of spiking in modeled MCs and sTCs. Histogram bars reflect mean ± SE. **(F)** Curves reflecting fits of a sigmoidal function (Eqtn 1 in Methods) to OSN stimulation intensity vs. simulated spike number data for each MC (*n* = 8, red) and sTC (*n* = 7, blue). **(G)** Values for the *stimulus*_50*%max*_ from fitted curves in part **(F)**. The smaller *stimulus*_50*%max*_ values for sTCs indicate that their spiking is more sensitive to OSN activity.

Within this framework, we quantified two aspects of the spiking behavior of MCs (*n* = 8) and sTCs (*n* = 7), the number of spikes and probability of spiking in a given trial, at each of four OSN stimulation levels. At all stimulus levels except 30 μA, sTCs had a significantly higher average number of spikes than MCs (Figure 4D; e.g., at 50 μA: 0.1 ± 0.1 spikes for MCs, 4.1 ± 1.0 spikes for sTCs; *p* = 0.0040, Mann-Whitney *U* test). sTCs also had a significantly higher spike probability at 50 μA (Figure 4E; 86 ± 14% for sTCs, 13 ± 9% for MCs; *p* = 0.0047, Mann-Whitney *U* test) and 100 μA (100 ± 0% for sTCs, 46 ± 17% for MCs; *p* = 0.0370, Mann-Whitney *U* test), but the spike probabilities converged to near 100% for both cells at 200 μA. These spiking characteristics are consistent with MCs having a reduced sensitivity vs. sTCs to similar levels of OSN activity.

The issue of sensitivity was also examined in the context of the relationship between stimulus intensity and the number of evoked spikes for individual MCs and sTCs. A sensitivity curve for each cell was generated by fitting a sigmoidal function (Equation 1 in Methods) to the stimulus intensity vs. spike number data for that cell (Figure 4F). This yielded a value for *stimulus*_50*%max*_ for spike number. Consistent with a lower sensitivity for MCs, we found that MCs had significantly higher *stimulus*_50*%max*_ values than sTCs (135 ± 19 μA, *n* = 8, vs. 70 ± 14 μA, *n* = 7; *p* = 0.0260, Mann-Whitney *U* test; Figure 4G).

The features of the modeled cells, the greater number of spikes and the higher spike probability with weaker stimuli for sTCs vs. MCs, mirror the properties of spiking of MCs and output tufted cells that have been observed *in vivo* in studies examining the odor concentration dependence of spiking (Igarashi et al., 2012; Kikuta et al., 2013). Some aspects of the *in vivo* spike responses were not recapitulated in our modeling. For example, the delay in spiking onset which is typically seen in MCs *in vivo* (Fukunaga et al., 2012; Igarashi et al., 2012) was not seen here. This was not surprising since this delay is likely at least partially due to inhibition (Fukunaga et al., 2012) which we did not include in this model.

### Differences in OSN Input and Cell Intrinsic Properties Mainly Contribute to the Greater Spiking in sTCs vs. MCs

Our analysis above suggested that MCs and sTCs differ in both the monosynaptic OSN and prolonged components of their excitatory currents, and these cells also have notable differences in intrinsic properties such as cell input resistance. To understand how these various properties contributed to the spike differences in the modeled MCs and sTCs, we exchanged each property between the modeled cell-types (Figures 5A,B) and then simulated their spiking responses (Figures 5C,D). We assessed whether any one exchange induced a statistically significant difference in spiking as follows. First, for each cell, we generated Mann-Whitney U statistic by comparing the values for the simulated spike numbers based on actual currents measured under the native condition to the spike numbers generated when we exchanged the component in question to that measured in the other cell-type (in all of the other cells). We then combined the Mann-Whitney U results for each of the cells with a Fisher Combined Test. This gave us a *p*-value for the probability that we would have observed the same effects or larger under a null model in which none of the cells truly had different responses with and without the exchange.

**Figure 5:** Use of NEURON simulations to determine cell parameters that impact spiking in MCs and sTCs. **(A)** Illustration of model MC and sTC used in our NEURON model, with input synapses shown in black. Differences in the length of lateral dendrites are not depicted although they were implemented in the model cells. **(B)** Color-coded table indicating the different cell-types that were modeled. Parameters that were varied included intrinsic properties (morphology and input resistance), the monosynaptic OSN-EPSC (“mono”), and the prolonged excitatory current. As an example, the magenta entry in the second line of the table corresponds to a cell with the intrinsic properties and prolonged currents of a MC but an OSN-EPSC of an sTC. **(C)** Single trial examples of simulated voltage responses for various versions of a MC shown in part **(B)** (50 μA OSN stimulation). Cells had either: **(i)** all MC parameters; **(ii)** all MC parameters, except a monosynaptic OSN-EPSC from sTCs (*MC*_*STCmono*_); **(iii)** all MC parameters except sTC prolonged current (*MC*_*STCpr*_); or **(iv)** MC OSN-EPSC and prolonged current, but intrinsic properties of sTCs (*MC*_*STCint*_). **(D)** Single trial examples of simulated voltage responses for various versions of the sTC shown in part **(B)** (50 μA OSN stimulation). **(E)** Summary of the change in the number of spikes that occurred upon exchanging the different excitatory current components and intrinsic properties between MCs and sTCs. Results are shown for MCs upon swapping in the sTC OSN-EPSC or prolonged current **(i)**; for sTCs upon swapping in the MC OSN-EPSC or prolonged current **(ii)**; and for both cell types upon swapping in the intrinsic properties of the other cell-type **(iii)**. There are many more data points than number of cells of each type (*n* = 8 for MCs, *n* = 7 for sTCs), reflecting the fact that for each trial for each cell, we swapped in the components measured in all of the other cells of the other cell-type. All results reflect data obtained at 50 μA OSN stimulation. **(F)** Spike probabilities measured for various versions of the MC **(i)** and sTC **(ii)** at 50 μA OSN stimulation. Each histogram bar reflects mean ± SE for that condition. Note that the only statistically significant difference was observed when we swapped in the intrinsic properties of the sTC while maintaining the excitatory currents of a MC (red and light blue histogram bars in **(Fi)**. In the spike probability measurements, we only made statistical comparisons between the “control condition” (e.g., the MC represented by the red bar in **Fi**) and one of the manipulated conditions (e.g., the MC with sTC intrinsic properties). Pair-wise comparisons between some of the other conditions (e.g., the MC with sTC prolonged currents vs. the MC with sTC intrinsic properties) may have revealed statistically significant differences, but the meaning of such differences would be ambiguous.

Using this approach, we found that the monosynaptic OSN conductance had a modest but significant impact on the number of spikes (Table 2 and Figures 5Ei,ii). At every stimulation intensity, substituting the OSN-EPSC in sTCs (*n* = 7 cells) into MCs (*n* = 8 cells) increased the number of spikes (e.g., at 50 μA: from 0.13 ± 0.07 to 0.50 ± 0.06, *p* = 0.025; Fisher Combined tests of Mann-Whitney *U* tests). This can be seen in the example traces in Figures 5Ci,Cii as a change from a non-spiking response (red trace = 0 spikes) to a response with 1 spike (magenta trace), as well as in the cluster of spike number-change values above zero for *MC*_*STCmono*_ in Figure 5Ei. Substituting the MC OSN-EPSC into sTCs had the opposite effect, decreasing the number of spikes at every stimulation intensity (e.g., 50 μA: from 4.05 ± 0.99 to 3.29 ± 0.34, *p* = 0.0003; Fisher Combined tests of Mann-Whitney *U* tests). This can be seen in the example traces in Figures 5Di,Dii as a change from 3 spikes (blue trace) to 2 spikes (teal trace), as well as in the cluster of spike number-change values below zero for *sTC*_*MCmono*_ in Figure 5Eii. In terms of spike probability, we found that substituting the monosynaptic OSN conductance changed the percent of trials showing a spike in some cells, but none of the observed changes were statistically significant (Table 3 and Figures 5Fi,ii).

**Table 2:** Values for the number of simulated spikes for modeled MCs and sTCs with various cellular properties exchanged.

**Stimulus intensity (μA)**	**MC (*n* = 8)**	**MC_**STCmon**_ (*n* = 8)**	**MC_**STCpr**_ (*n* = 8)**	**MC_**STCint**_ (*n* = 8)**	**sTC (*n* = 7)**	**sTC_**MCmonor**_ (*n* = 7)**	**sTC_**MCpr**_ (*n* = 7)**	**sTC_**MCint**_ (*n* = 7)**
30	0.08 ± 0.08	0.50 ± 0.06 *p* = 0.0058	0.15 ± 0.04 *p* = 0.4050	9.89 ± 1.56 *p* < 0.0001	1.71 ± 0.84	1.14 ± 0.10 *p* = 0.0001	10.57 ± 1.12 *p* = 0.0220	0.51 ± 0.11 *p* < 0.0001
50	0.13 ± 0.09	0.50 ± 0.06 *p* = 0.0245	0.30 ± 0.05 *p* = 0.1664	11.83 ± 1.91 *p* < 0.0001	4.05 ± 0.99	3.29 ± 0.34 *p* = 0.0003	12.59 ± 1.28 *p* = 0.0232	0.67 ± 0.13 *p* < 0.0001
100	0.71 ± 0.36	1.15 ± 0.10 *p* = 0.0001	0.91 ± 0.16 *p* = 0.0105	18.93 ± 2.43 *p* < 0.0001	12.10 ± 5.22	11.35 ± 1.21 *p* = 0.0106	19.68 ± 1.57 *p* < 0.0001	1.32 ± 0.29 *P* < 0.0001
200	4.58 ± 3.40	5.68 ± 0.71 *p* = 0.0044	1.76 ± 0.20 *p* = 0.0001	37.25 ± 4.21 *p* < 0.0001	15.38 ± 4.76	13.33 ± 1.06 *p* < 0.0001	39.80 ± 2.56 *p* < 0.0001	2.47 ± 0.39 *p* < 0.0001

*As in Figure 5, three cellular properties were varied: the monosynaptic OSN-EPSC, the prolonged excitatory current, and cell intrinsic properties. Cell-type is indicated by a notation X_Y_, where X is the cell-type (MC or sTC) that contributes two of the three properties and Y indicates the swapped-in property from the other cell-type. Thus, for example, MC_STCmono_ indicates a cell that had the prolonged currents and intrinsic properties of a MC but the monosynaptic OSN-EPSC of an sTC. Values in the table reflect mean ± SE. The n values in the top row reflect the number of experimental recordings; in each recording, all four OSN stimulation intensities were sampled. The p values reflect the results of application of the Fisher Combined statistical test across all experimental recordings comparing the control condition (all-MC or all-sTC) with each of the indicated manipulated conditions (see Methods)*.

**Table 3:** Spike probability (%) values for modeled MCs and sTCs with various cellular properties exchanged.

**Stimulus intensity (μA)**	**MC (*n* = 8)**	**MC_**STCmono**_ (*n* = 8)**	**MC_**STCpr**_ (*n* = 8)**	**MC_**STCint**_ (*n* = 8)**	**sTC (*n* = 7)**	**sTC_**MCmono**_ (*n* = 7)**	**sTC_**MCpr**_ (*n* = 7)**	**sTC_**MCint**_ (*n* = 7)**
30	8 ± 8 %	34 ± 4% *p* = 0.5077	9 ± 2% *p*=0.9944	61 ± 5% *p*=0.0341	52 ± 19%	53 ± 6% *p* = 0.9973	75 ± 4% *p* = 0.6763	33 ± 6% *p* = 0.8842
50	13 ± 9	34 ± 6 *p* = 0.9478	22 ± 5 *p* = 0.5629	62 ± 5 *p* = 0.0341	86 ± 14	82 ± 4 *p* = 0.9673	83 ± 4 *p* = 0.8374	36 ± 6 *p* = 0.2509
100	46 ± 17	67 ± 5 *p* = 0.3720	35 ± 5 *p* = 0.8640	99 ± 1 *P* = 0.0854	100 ± 0	94 ± 3 *p* = 1	100 ± 0 *p* = 1	51 ± 7 *p* = 0.2509
200	88 ± 13	86 ± 4 *p* = 0.9478	76 ± 5 *p* = 0.8640	100 *P* = 0.9478	100 ± 0	100 ± 0 *p* = 1	100 ± 0 *p* = 1	82 ± 5 *p* = 1

*Same notation and statistical parameters as Table 2. Note that there were only a few exchanges that caused statistically significant differences in spike probability*.

Exchanging the prolonged current component of MCs and sTCs significantly impacted spiking in our model cells, but not in a manner that would explain sTCs' greater spiking sensitivity (Figure 4). Substituting the MC prolonged signal into sTCs *increased* the number of spikes at every stimulus intensity (e.g., 50 μA: from 4.05 ± 0.99 to 12.59 ± 1.28; *p* = 0.023; Fisher Combined test of Mann-Whitney *U* tests; Table 2 and Figures 5Di,Diii and Figure 5Eii), while substituting the sTC prolonged signal into MCs had the opposite effect on spike number, at least at the highest 200 μA intensity (from 4.58 ± 1.89 to 1.76 ± 0.02; *p* = 0.0001, Fisher Combined test of Mann-Whitney *U* tests; Table 2). These effects were consistent with the generally larger size and longer-lasting prolonged current in MCs vs. sTCs (Figure 3). These results indicate that sTCs spike more than MCs *in spite* of MCs having larger prolonged currents.

Our final analysis examined the contribution of the intrinsic properties of MCs and sTCs, including morphology and input resistance, on the cells' spiking characteristics. This was done by fixing the monosynaptic OSN and prolonged components of a given cell's excitatory current input while substituting the intrinsic properties with those of the other cell type. The intrinsic properties that we substituted were resistance per unit area (estimated from our experimentally measured input resistance values), the cellular morphology, and resting potential (see Methods and Table 1). We found that substituting MC intrinsic properties into sTCs (*sTC*_*MCint*_) led to a significant decrease in the number of spikes at every stimulus intensity (e.g., 50 μA: from 4.05 ± 0.99 to 0.67 ± 0.13; *p* < 0.0001; Fisher Combined test of Mann-Whitney U tests; Figures 5Di,iv and Figure 5Eiii and Table 2), while substituting sTC intrinsic properties into MCs increased the number of spikes (e.g., 50 μA: from 0.13 ± 0.09 to 11.83 ± 1.91; *p* < 0.0001; Fisher Combined test of Mann-Whitney *U* tests; Figures 5Ci,iv and Figure 5Eiii and Table 2). Substituting sTC intrinsic properties into MCs also increased the probability of spiking at the two lower stimulation intensities (e.g., at 50 μA: from 12.5 ± 8.8% to 61.9 ± 5.3%; *p* = 0.0340; Fisher Combined test of Mann-Whitney *U* tests; Figure 5Fi and Table 3). Our analysis of cell intrinsic properties focused on the passive properties of the cells and did not take into factors such as potential differences in voltage-gated ion channels between MCs and TCs (Liu and Shipley, 2008; Burton and Urban, 2014). However, our results indicate that passive properties such as cell input resistance at least partially explain the spiking differences between MCs and sTCs.

### Functional Advantage of Having Two Populations of Output Neurons With Distinct Stimulus-Response Relationships

Our results above have shown that MCs and sTCs display differences in their stimulus-response relationship and also identified mechanisms that could underlie this difference. The difference in the stimulus-response relationship was most clearly reflected in the rightward shifts in the relationship between OSN stimulation intensity and number of simulated spikes for individual MCs/sTCs (Figures 4F,G). For information processing, what might be the value of having two types of output cells with differing stimulus-response relationships?

One way to answer this question is to consider the sensitivity of MCs and sTCs to changes in OSN stimulation intensity. This sensitivity, as reflected in the slope of a stimulus-response curve, indicates how effectively the population of MCs and sTCs carries information about changes in OSN activity through changes in spiking rates. To evaluate the added advantage of having two output cell populations to this effectiveness, we first derived average stimulus response curves for two scenarios, one (Condition A) in which we assumed that the MC and sTC populations each individually carried information about the level of OSN activity (the actual situation) and a second (Condition B) in which we grouped all MCs and sTCs into one population with a stimulus-response relationship that was average between that of MCs and sTCs. The stimulus-response curves were generated from the sigmoidal curves that were fitted to the OSN stimulation intensity vs. spike number data for individual MCs/sTCs (Figures 4F,G), either averaging them for all cells of a given cell-type (the blue and red curves in Figure 6A) or across all cells of both types **(**black curve in Figure 6A). Then, to measure the sensitivity of the cell populations in the two scenarios, we calculated the square of the derivative of the stimulus-response curves for the two conditions. As can be seen in Figure 6B, the cell population in Condition A displayed a greater sensitivity at most stimulus intensities vs. Condition B, and also was sensitive to a wider range of stimulus strengths. Thus, two populations of output neurons with distinct stimulus-response relations are more effective at carrying information about changes in stimulus strength than a single population of output neurons.

**Figure 6:** Two populations of output cells with distinct stimulus-response relations better report changes in OSN activity. **(A)** Comparison of stimulus response curves under scenarios in which MCs and sTCs have distinct sensitivities to OSN activity (Condition A) vs. if there were only a single population of output cells with a sensitivity that was the average of MCs and sTCs (Condition B). The curves representing Condition A reflect the average behavior of all test cells within our MC population (red) and the average of all test cells within our sTC population (blue). Condition B is reflected by the black curve. The stimulus-response for each cell was the sigmoidal curve fitted to the OSN stimulation vs. simulated spike number data for that cell (see curves in Figure 4F). **(B)** Sensitivity measurement for Condition A (purple) and Condition B (black). Each curve was generated by taking the squared derivative of the stimulus response curve for each cell under the two conditions and averaging that across all cells (see Methods). The larger values for Condition A at low and high stimulation intensities indicate that two populations of cells with distinct sensitivities more effectively report changes in OSN activity than a single population of cells.

It should be noted that our analysis, which was based on the average behavior of MCs and sTCs for both Conditions A and B, ignored cell-to-cell variabilities within the subpopulation of MCs or sTCs. Such variance in the stimulus-response relationships for individual MCs or sTCs can be observed in the different positions along the x-axes for the fitted sigmoidal curves in Figure 4F. We chose to ignore the within-cell type variance in order to simplify our analysis of the contribution of differently-behaving cell-types to the information carrying capacity of the network of bulb output neurons.

## Discussion

In this study, we combined experimental and computational methods to examine mechanisms that could contribute to differences in the spiking properties of different populations of excitatory neurons in the olfactory bulb. The principal focus was on MCs and a subpopulation of output TCs, the sTCs. Our main findings in our comparison between MCs and sTCs were that: (1) sTCs have a number of differences in their excitatory currents from MCs, including larger direct OSN input currents but smaller prolonged currents; (2) sTCs are more sensitive than MCs, producing more spikes at lower levels of OSN activity; (3) the greater spiking in sTCs reflects both the greater OSN input signals as well as differences in their intrinsic properties; and (4) differences in sensitivity of sTCs vs. MCs enhances the ability of the bulb to encode changes in stimulus intensity. We also characterized experimentally a number of novel properties of the excitatory currents of another class of TCs, the eTCs. These points are discussed below.

### Mechanisms That Contribute to Different Spike Sensitivities of MCs and Output TCs

Recent physiological studies *in vivo* have indicated that MCs and TCs have markedly different responses to odors. MCs require higher concentrations of an odorant to be activated, displaying rightward-shifted odor-concentration vs. spike response curves (Igarashi et al., 2012; Kikuta et al., 2013). MCs also appear to have a narrower odor tuning profile than TCs (Nagayama et al., 2004; Kikuta et al., 2013). Because any one odorant receptor that is associated with a glomerulus can bind to multiple types of odors with varying affinities, the narrower odor tuning of MCs likely reflects similar mechanisms as the rightward-shifted odor concentration vs. activation curves. To understand potential mechanisms that contribute to spiking differences between MCs and sTCs, we took a two-pronged approach, first using whole-cell patch-clamp recordings in bulb slices to compare the basic electrophysiological properties of MCs and sTCs. This was followed by computational modeling, in which we used a component-swapping approach to assess the contribution of the different cellular aspects recorded experimentally to spiking differences. Our analysis revealed that the greater sensitivity of sTCs vs. MCs was due both to the sTCs' ~2-fold larger direct OSN input current (the OSN-EPSC) as well as intrinsic properties such as their much higher input resistance. Importantly, prior to exchanging the electrophysiological aspects in MCs/sTCs in our modeling, we were able to reproduce the greater spiking sensitivity of TCs vs. MCs that has been observed *in vivo* (Griff et al., 2008; Fukunaga et al., 2012; Igarashi et al., 2012; Kikuta et al., 2013) when we input our experimentally-measured currents into the model cells (Figure 4). This helped to validate our brain slice and computational techniques as an approach to investigate *in vivo* differences between MCs and TCs.

Our study adds to a growing literature that has examined the mechanistic basis for differing odor-evoked spike responses in MCs vs. TCs. In one such study, conducted by Burton and Urban (2014), the authors concluded, as we did, that the greater spiking sensitivity in TCs reflected a combination of stronger OSN input drive as well as greater intrinsic excitability. However, our study differed from theirs in a number of ways, including in the subtypes of TCs that were examined. While we analyzed sTCs, Burton and Urban (2014) mainly focused on mTCs. Our choice to focus on sTCs was based on the fact that sTCs are the most morphologically distinct from MCs of all TC subtypes. In addition, previous *in vivo* analysis (Griff et al., 2008) has suggested that TCs near the border between the EPL and the glomerular layer—presumably sTCs as we have defined them—display much more dramatic differences in their odor-evoked responses from MCs as compared to mTCs. Our study was also unique in that it examined MC/sTC responses to a widely varying OSN stimuli. This approach allowed us to make more direct conclusions about the causes of the rightward-shifted odor concentration vs. spike response curves that have been observed *in vivo* for MCs vs. TCs. For example, we found in our analysis that many of the largest changes in spike number and probability upon exchanging the MC/sTC components occurred at low OSN stimulation intensities, when sTCs but not MCs were significantly active. This argued that the specific components in question contributed to shifts in the activation curves.

There are naturally caveats associated with the fact that our analysis of MCs and sTCs was conducted *in vitro* rather than *in vivo*. Perhaps chief amongst them was the nature of the stimulus. While an odor activates OSNs in a distributed fashion over the duration of a sniff, we examined responses to a single electrical stimulus pulse applied to OSN axons. A priori, it is not clear whether this difference in stimuli should impact any of our fundamental conclusions about what underlies the spike differences in MCs and sTCs, but it is nevertheless a notable limitation of our study. At the same time, our *in vitro* approach using a discrete stimulus applied locally to OSNs offered the advantage of a much-simplified system in which we could largely ignore the contribution of interglomerular interactions and centrifugal feedback mechanisms on spike differences between MCs and sTCs. This enabled us to focus on the impact of local excitatory mechanisms and cell intrinsic properties on the spike differences. There are certainly a number of cellular and synaptic mechanisms that we did not examine that could contribute to spiking differences between MCs and sTCs in addition to the ones we identified. For example, differences in GABAergic inhibition are already known to contribute to spike timing differences between MCs and some TCs (Fukunaga et al., 2012; Geramita et al., 2016; Burton et al., 2017; Geramita and Urban, 2017). In comparing MCs and sTCs in particular, the much shorter lateral dendrites of sTCs should mean that sTCs are less impacted than MCs by long-range interglomerular interactions mediated by granule cells. This may contribute to sTCs more faithfully reporting odor-evoked activation of OSNs at their target glomerulus than MCs.

### Cellular and Synaptic Mechanisms of MCs, sTCs, and eTCs

Besides providing insight into mechanisms underlying spiking differences between MCs and sTCs, our study also provided a number of novel insights into the basic cellular and synaptic properties of various excitatory bulbar neurons. First, we extended the available information about what is known about differences in OSN-EPSCs between MCs and eTCs, which are a class of glutamatergic interneurons that reside in the glomerular layer. Prior reports have shown that, at least at some OSN stimulation intensities, the OSN-EPSC in eTCs is much larger than in MCs (Najac et al., 2011; Gire et al., 2012; Vaaga and Westbrook, 2016). The very large OSN signal in eTCs is functionally important, since it causes eTCs to spike at much lower levels of OSN activity than MCs and also contributes to eTC-mediated feedforward excitation dominating the MC response to OSN stimulation (De Saint Jan et al., 2009; Gire et al., 2012; Vaaga and Westbrook, 2016). Here, we found that the OSN-EPSC in eTCs was ~5-fold larger than in MCs at high OSN stimulation intensities, when all OSN axons at the target glomerulus were presumably active, and, also, that a major contributor to this difference was a much larger “unitary” EPSC in eTCs driven by each OSN axon. Perhaps the most striking result in this respect for MCs was the extremely low frequency of spontaneous EPSCs (sEPSCs) that in part reflect spike activity in single OSNs. The low frequency likely was due to the fact that most sEPSCs were so small that they were buried in recording noise. Because morphological analyses has suggested that OSNs form a similar number of OSN synapses onto MCs and eTCs (Bourne and Schoppa, 2017), we attribute the very small sEPSCs in MCs to the unusual physiological properties of the MC apical dendrite, for example the high density of gap junctions (Christie et al., 2005; Pimentel and Margrie, 2008) that may filter direct OSN input signals (Gire et al., 2012). What might contribute to the 2-fold difference in size of the OSN-EPSC between MCs and sTCs at high OSN stimulation intensities (see above)? In this study, we attempted to address this question by recording unitary EPSCs in MCs and sTCs, but the small size of these events in both cells made a comparative analysis difficult.

We also characterized more prolonged excitatory currents that are evoked by OSN stimulation across MCs, sTCs, and eTCs. Interestingly, we found that sTCs stood out from MCs and eTCs in the small magnitude of the prolonged currents, especially in a sustained component that persisted for hundreds of milliseconds after OSN stimulation. The sustained evoked current, at least in MCs, reflects activation of Group I mGluRs (Schoppa and Westbrook, 2001; Heinbockel et al., 2004; Ennis et al., 2006; Yuan and Knöpfel, 2006; De Saint Jan and Westbrook, 2007), while eTCs are known to support large Group I mGluR-mediated currents that reflect the opening of Ca2+-activated non-selective cation channels (Dong et al., 2009). Our results thus suggest that sTCs may differ from other excitatory neurons in the bulb in their low expression of Group I mGluRs or weak coupling of the receptors to cation channels. In terms of impact on spike activity, we found in our modeling that the smaller prolonged excitatory currents in sTCs were not a major contributor to the higher spiking sensitivity of sTCs. Indeed, in our component-swapping computational analysis, we found that replacing the sTCs' prolonged current with that of MCs increased spiking, suggesting that sTCs spike more than MCs in spite of their weak prolonged current signals.

It should be noted that there were some sources of uncertainty in the analysis of the prolonged excitatory current components. For example, the extracellular solution in which the slow currents were recorded did not include added glycine, which is a co-agonist for NMDA receptors. Because slow excitation of at least MCs partially depends on NMDA receptors (Carlson et al., 2000; Schoppa and Westbrook, 2001), the absence of added glycine may have impacted our estimates of the magnitude of slow excitation. However, we do not believe that this was a significant cause of error. Other studies examining slow excitation (Carlson et al., 2000; Schoppa and Westbrook, 2001) have shown robust NMDA receptor-mediated activation of MCs in the absence of added glycine, suggesting that there is significant residual glycine in the slice. In addition, for our conclusion to be wrong – that the slow current is larger in MCs/eTCs than in sTCs—it would require that the absence of glycine had differential effects on the slow currents in the different cell types. This, we believe, is unlikely.

### Broader Implications for Information Processing

A final issue that we addressed in our study was what broader function might be served by having two classes of output cells in the bulb with differing sensitivities to OSN activity (Igarashi et al., 2012; Kikuta et al., 2013). In our study, this difference in sensitivity was perhaps best seen as a rightward shift in the OSN stimulation vs. spike response curve in MCs vs. sTCs (Figures 4F,G). We addressed this question here quite simply by comparing the steepness of the OSN stimulation intensity vs. spiking curves that we observed in MCs and sTCs with that produced in a hypothetical situation in which bulbar output was carried by a single population of cells with an activation profile that reflected the average between that of MCs and sTCs. This analysis revealed that having two populations of output cells with distinct stimulus-response relations enabled the bulb to better report small changes in OSN activity. In terms of olfactory behavior, we would suggest that this enhanced coding capability would directly impact the ability of an animal to discriminate different concentrations of odors (Geramita et al., 2016) and/or help in the discrimination of different but similar odors that produce small differences in OSN activity at a specific glomerulus. It should be noted that, while our functional analysis included two classes of output cells, MCs and sTCs, it did not include mTCs. Because mTCs have morphological features that are intermediate between that of MCs and sTCs, it is tempting to speculate that mTCs could report OSN activity changes in a range that is intermediate between MCs and sTCs. mTCs could thus further amplify an animal's ability to discriminate small odor concentration differences or structurally similar odors. In this context, it is notable that in our sensitivity analysis (Figure 6B), there was an intermediate OSN stimulus range in which our model that included only one population of “hybrid” MC/sTCs cells performed somewhat better at coding changes in OSN activity than our model with differently-behaving MCs and sTCs. Perhaps this intermediate range is mainly coded by mTCs.

Amongst sensory systems, the olfactory bulb is hardly unique in having multiple types of output cells that provide parallel pathways for information flow. Such pathways are perhaps best characterized in the retina where there are at least 30 types of ganglion cells each with distinct tuning to visual stimuli (Masland, 2012; Sanes and Masland, 2015; Baden et al., 2016). Some of the different classes of ganglion cells report the same stimulus but with different intensity thresholds (Kastner and Baccus, 2011) in much the same way that MCs and TCs appear to do for odorant stimuli (Kikuta et al., 2013). The presence of different populations of ganglion cells maximizes the transmission of highly accurate information about visual stimuli to the lateral geniculate nucleus (Segev et al., 2006; Kastner et al., 2015). There are however some important mechanistic differences between how the parallel pathways for information flow are generated across sensory systems. In many sensory structures, the different response properties of the output cells often simply reflect differences in the initial stages of stimulus detection that are then maintained through selective feedforward connections. However, in the bulb, it is very unlikely that MCs and TCs at the same glomerulus receive input from distinct types of OSNs. Thus, response differences between MCs and TCs must arise due to cell intrinsic properties and synaptic connections within the bulb.

## Data Availability Statement

The raw data supporting the conclusions of this article will be made available by the authors, without undue reservation.

## Ethics Statement

The animal study was reviewed and approved by Institutional Animal Use and Care Committee, University of Colorado, Anschutz Medical Campus.

## Author Contributions

SJ, JZ, and NS: design of experiments, interpretation of results, and writing of manuscript. SJ: acquisition and analysis of data. All authors contributed to the article and approved the submitted version.

## Conflict of Interest

The authors declare that the research was conducted in the absence of any commercial or financial relationships that could be construed as a potential conflict of interest.
